RETRACTED

# Efficacy of Fuyuan Xingshen Decoction Combined with Butylphthalide Sodium Chloride Injection in the Treatment of Acute Cerebral Infarction and Its Effect on Hemodynamics

**DOI:** 10.1155/2022/2402040

**Published:** 2022-09-19

**Authors:** Jiangang Ji, Kai Yu, Xinyu Zhang, Wenting Liu

**Affiliations:** ^1^Department of Encephalopathy, Weifang Traditional Chinese Hospital, Weifang, Shandong 261041, China; ^2^Department of Neurology, Weifang People's Hospital, Weifang, Shandong 261041, China

## Abstract

**Objective:**

This study aims to determine the curative effect of Fuyuan Xingshen Decoction combined with butylphthalide sodium chloride injection in acute cerebral infarction (ACI) treatment and its effect on hemodynamics.

**Methods:**

In our hospital, a total of 84 ACI patients from May 2020 to February 2022 were randomly divided into two groups: observation and control (*n* = 42 each). Fuyuan Xingshen Decoction in combination with butylphthalide sodium chloride injection was provided to the observation group, while the control group received butylphthalide sodium chloride injection alone. Both groups' clinical efficacy was observed. Before and after treatment, the neurological function of the two groups was evaluated using the National Institutes of Health Stroke Scale (NIHSS), while the daily living ability of both groups was determined using the Barthel index rating scale. Both groups were investigated for their cognitive function, before and after treatment, by using the Mini-Cog scale and Montreal Cognitive Assessment (MoCA) scale. The pulsatility index (PI), peak velocity (Vp), and mean velocity (Vm) of intracranial arteries were measured by transcranial Doppler ultrasonography before and after treatment. The levels of ubiquitin carboxy-terminal hydrolase-1 (UCH-L1), Fibulin-5, and visinin-like protein-1 (VILIP-1) in serum and the expression levels of miR-34c, miR-25, and miR-182 in peripheral blood of the two groups were compared. Both groups were observed for the incidence of adverse reactions.

**Results:**

Compared with the control (71.43%), the observation group exhibited a significantly higher effective rate of around 90.48%. In the observation group, the improvement in NIHSS, Barthel index, Mini-cog, and MoCA scores; hemodynamic indexes including Vp, PI, and Vm; serum UCH-L1, Fibulin-5, and VILIP-1 levels; and the miR-34c, miR-25, and miR-182 expression levels in peripheral blood was better than the control group, with significant difference (all *P* < 0.05). The incidence of adverse reactions between the groups demonstrated no significant differences (*P* > 0.05).

**Conclusions:**

Fuyuan Xingshen Decoction combined with butylphthalide sodium chloride injection can effectively improve patients' daily living ability, neurological function, cognitive function, and cerebral hemodynamics in the treatment of ACI, with good effect and safety.

RETRACTED

## 1. Introduction

Acute cerebral infarction (ACI) is a kind of common acute brain disease. It is the pathological necrosis of brain tissue caused by sudden reduction or interruption of blood flow in the local artery and insufficient oxygen and blood supply to local brain tissue. The pathogenesis of cerebral infarction is complex, which is related to apoptosis, inflammatory response, free radical damage, and other mechanisms. This disease can easily lead to disability or death, and most patients with ACI will suffer from impaired work ability, language dysfunction, and motor dysfunction [1, 2]. Epidemiological studies show that there are 1.5–2 million new stroke cases in China every year and more than 7 million cases of existing cerebrovascular disease patients. Cerebral infarction accounts for about 70% of cerebrovascular diseases [3]. The pathophysiological change of cerebral infarction is a complicated process, and it is difficult to achieve a good effect with a single drug treatment for brain tissue and nerve function damage. Currently, surgical thrombectomy and drug thrombolysis are the most common clinical therapies for ACI. For those patients who exceed the time window of thrombolysis or are not suitable for thrombolysis and thrombectomy for various reasons, the combination of Western and Chinese medicine can be used to improve the microcirculation of cerebral blood flow. Butylphthalide sodium chloride injection is a common clinical medicine for cerebral infarction, which has a good therapeutic effect in many pathological links of cerebral infarction. The drug can improve the circulation of ischemic cerebral tissue, promote cerebral angiogenesis, increase collateral blood flow in the infarcted area, and ultimately improve cerebral nerve function [4]. According to traditional Chinese medicine, positive Qi deficiency and the complication of wind-phlegm and stagnant heat are the pathogenesis of cerebral infarction. The method of reviving energy method can strengthen essence while dispelling the wind, and it can rest the wind while awakening the mind [5]. This study aims to investigate the efficacy of Fuyuan Xingshen Decoction combined with butylphthalide sodium chloride injection in the treatment of ACI and its effect on hemodynamics.

## 2. Materials and Methods

### 2.1. General Data

A total of 84 patients who were diagnosed with ACI and received treatment at our hospital between May 2020 and February 2022 were randomly divided into two groups: an observation and a control group (*n* = 45 each). The observation group included a total of 23 males and 19 females, between 45 and 75 years of age. The average age of the group was 59.17 ± 7.31 years. The time from beginning to admission ranged from 1 to 21 h, with an average time of 14.12 ± 5.85 h. There were 13 cases of hyperlipidemia, 17 cases of hypertension, and 10 cases of diabetes that resulted from the complications. Cerebral infarction sites included basal ganglia in 14 cases, para-somatic lateral ventricles in 7 cases, thalamus in 18 cases, and other sites in 3 cases. The control group included 27 males and 15 females ranging in age from 44 to 74 years old, with an average age of 59.39 ± 5.54 years. The time from beginning to admission ranged from 2 to 24 h, with an average of 14.40 ± 6.16 h. Complications included 15 cases of diabetes, 12 cases of hypertension, and 9 cases of hyperlipidemia. Cerebral infarction sites included basal ganglia in 17 cases, para-somatic lateral ventricles in 4 cases, thalamus in 20 cases, and other sites in 1 case. General findings were comparable between the groups (*P* > 0.05). The hospital's ethics committee approved this study.

RETRACTED

### 2.2. Inclusion Criteria

The following are the inclusion criteria: (1) all patients met the diagnostic criteria of *“Guidance on The Diagnosis and Treatment of Cerebral Infarction with Integrated Traditional Chinese and Western Medicine (2017)”* [6] and were confirmed by imaging examination; (2) all patients were in line with the wind-phlegm obstruction syndrome in the “Guidelines for Clinical Research on New Chinese Medicine (Trial)” [7], and the primary symptoms were hemiplegia, askew tongue, and sensory subsided while the secondary symptoms were dizziness, dark tongue, white tongue coating, and slippery pulse; (3) the onset time was within 72 h; (4) all cases were the first onset; (5) all patients participated in this study voluntarily; and (6) the family members agreed to the patient's participation in this study.

### 2.3. Exclusion Criteria

The following are the exclusion criteria: (1) patients with obvious intracranial hemorrhage; (2) patients who were preparing to receive or had received thrombolytic treatment; (3) patients having severe organ dysfunction, including those of the heart, liver, and kidneys; (4) patients suffering from a mental disorder or consciousness dysfunction; (5) patients allergic to the drugs; (6) patients with coagulation dysfunction; (7) patients who are going to receive or have received surgical thrombectomy; and (8) comatose or unconscious patients.

### 2.4. Methods

In both groups, anticoagulation, respiratory support, reduction of intracranial pressure, correction of water and electrolyte, lipid-lowering, depressurization, glucose control, and other traditional therapies were administered. The control group was given butylphthalide sodium chloride injection (EBP Pharmaceutical Co., LTD., Shijiazhuang Pharmaceutical Group, SFDA approval number: H20100041), and the drug was given intravenously at 100 ml/time, twice a day. The observation group received Fuyuan Xingshen Decoction in accordance with the prescription of the control group. The recipe composition was: *Codonopsis pilosula* 30 g, *Leonurus japonicus* 30 g, Rhizomaacorigraminei 12 g, pseudo-ginseng 10 g, leeches 10 g, rhubarb 10 g, and Rhizomaarisaematis 15 g, all decocted in the hospital traditional Chinese medicine (TCM) pharmacy. According to the standard of 200 ml/time, twice/day, 14 d as a course, both groups were continuously treated for 14 d. The control group was supplemented with the same volume of normal saline to ensure a single variable.

RETRACTED

### 2.5. Observational Indices

(1) Clinical efficacy. (2) NIHSS, Barthel index, Mini-cog, and MoCA scores. The National Institutes of Health Stroke Scale (NIHSS) [8] with scores ranging from 0 to 45 was utilized for the assessment of the neurological function of the groups before and after treatment. The higher the score, the greater the severity of the neurological deficit. The Barthel index rating scale [9] was used to assess the two groups' daily living ability, with a range of total scores from 0 to 100. The higher the score, the higher the patients' daily living ability. The Mini-cog and MoCA scales [10] were used to measure the cognitive function of the two groups prior to and following treatment. The total score of Mini-cog ranged from 0 to 30. The MoCA scale included 11 items from 8 dimensions, and 30 points were the total score. The higher the score, the greater the state of cognitive function. Scorings were done by fixed staffs and the principle of blinding was adopted. (3) Hemodynamic indices. The peak velocity (Vp), the mean velocity (Vm), and the pulsatility index (PI) of intracranial arteries were evaluated by transcranial Doppler ultrasonography before and after treatment. (4) Serum biochemical indices. Before and after treatment, 10 mL of blood was collected from the veins in both groups. While the subjects were fasting in the morning, blood samples were collected and divided into two procoagulant test tubes. One blood sample's upper layer was extracted, deposited in a centrifuge tube, and centrifuged for 15 min at 3000 r/min with a 10 cm radius. For testing, the upper layer of serum was collected and kept at −70°C. The levels of ubiquitin carboxy-terminal hydrolase-1 (UCH-L1) and Fibulin-5 were evaluated using a double-antibody sandwich chemiluminescence assay, and the level of visinin-like protein-1 (VILIP-1) in serum was assessed using an enzyme-linked immunosorbent assay (ELISA). The instrument was an AxSYM chemiluminescence analyzer (Abbott, USA), and the kit was purchased from R&D company (USA). All procedures were operated according to the kit instructions. (5) miRNA level in peripheral blood. Total RNAs were extracted from the collected peripheral blood using Trizol. The first strand of cDNA was produced using a reverse transcription kit, and real-time PCR was carried out utilizing the CFX 96 qPCR detection system. The reaction conditions were set such that denaturation was carried out at 95°C for 5 s, followed by annealing for 30 s at 60°C, for a total of 40 cycles. The miR-34c, miR-25, and miR-182 expression levels in peripheral blood were determined. (6) Occurrence of adverse reactions.

RETRACTED

### 2.6. Efficacy Evaluation Criteria

The two groups' clinical efficacy was assessed using the *Diagnostic Efficacy Assessment Criteria for Stroke* [11]. Clinical recovery: after treatment, NIHSS of patients decreased by ≥90% compared with that before treatment, and the degree of disability was grade 0. Markedly effective: NIHSS was decreased by 46%∼89% after treatment, and grade 1∼3 was the degree of disability. Effective: After treatment, NIHSS was reduced by 21%∼45%, and the degree of disability remained unchanged. Ineffective: NIHSS decreased by <21% after treatment, and the degree of disability remained unchanged or worsened. Total effective rate = clinical recovery rate + markedly effective rate + effective rate.

### 2.7. Statistical Methods

All data in this survey were inputted into Excel form by two people without communication and processed by statistical software SPSS24.0. The measurement data were expressed as Mean ± SD ($\bar{x}\pm S$), and the *T*-test was adopted when the data were in line with normal distribution and the variance was uniform. The counting data were described by *n* and %, and the chi-squared test was used for intergroup comparison. Comparison of disordered classification data used the chi-squared test or Fisher's exact probability method, both of which were two-sided tests. *P* < 0.05 was considered as a statistically significant difference.

## 3. Results

### 3.1. Comparative Analysis of the Clinical Efficacy of the Two Groups

The total effective rate was significantly higher in the observation group (90.48%) than in the control group (71.43%; *P* < 0.05, Table 1).

### 3.2. Comparative Analysis of NIHSS, Barthel Index, Mini-Cog, and MoCA Scores between the Groups before and after Treatment

Prior to the administration of the treatment, the NIHSS, Barthel index, Mini-cog, and MoCA scores in the two groups were not significantly different from one another (all *P* > 0.05). Following treatment, the NIHSS score increased in both groups, although the Barthel index, Mini-cog, and MoCA scores decreased. In the observation group, scores on the NIHSS, Barthel index, Mini-cog, and MoCA improved more than in the control group (all *P* < 0.05, Table 2).

RETRACTED

### 3.3. Comparative Analysis of the Two Groups' Hemodynamic Indices before and after Treatment

Prior to the administration of the treatment, the levels of Vp, PI, and Vm in the two groups were not significantly different from one another (all *P* > 0.05). Following the administration of the treatment, the levels of Vp and Vm increased, although the level of PI dropped in both groups. However, the degree to which Vp, PI, and Vm improved in the observation group was significantly higher as compared to the control group (all, *P* < 0.05, Table 3).

### 3.4. Comparative Analysis of the Serum Levels of UCH-L1, Fibulin-5, and VILIP-1 between the Groups before and after Treatment

Prior to treatment, the levels of UCH-L1, Fibulin-5, and VILIP-1 did not exhibit a significant difference between the groups (all *P* > 0.05). Following treatment, serum UCH-L1, Fibulin-5, and VILIP-1 levels decreased in both groups, and the improvement degree of serum UCH-L1, Fibulin-5, and VILIP-1 was greater in the observation group than in the control group (all *P* < 0.05, Table 4; Figures 1–3).

### 3.5. Comparative Analysis of the miR-34c, miR-25, and miR-182 Expression Levels in Peripheral Blood before and after Treatment in the Two Groups

Peripheral blood levels of miR-34c, miR-25, and miR-182 were not significantly different between the groups prior to the treatment (all *P* > 0.05). MiR-25 expression increased in both groups following treatment, while miR-34c and miR-182 expression levels dropped in both groups. While in the observation group, greater improvement of miR-34c, miR-25, and miR-182 expression levels in peripheral blood was observed as compared to the control group (all *P* < 0.05, Table 5; Figures 4–6).

### 3.6. Comparative Analysis of Adverse Reactions between the Groups

In terms of the occurrence of adverse reactions, no difference could be considered statistically significant between the groups (*P* > 0.05, Table 6).

## 4. Discussion

ACI is classified as a “stroke” in TCM and is caused by a lack of good Qi. Its main pathogenesis is the mutual blocking of wind, phlegm, and stasis. When the patient suffers from an internal injury due to fatigue, or the spleen and stomach are damaged by fat, sweet, thick, and greasy things, it is easy to lead to spleen and stomach injury and eventually lead to the loss of healthy operation of the spleen, weakness of the spleen and stomach, and dereliction of duty in transportation and transformation. The stagnant body fluid can gather to form phlegm. The phlegm is turbid and intrinsic. The phlegm and dampness condense in the pulse, and the movement of Qi and blood will be blocked. The interaction of phlegm and blood stasis will lead to disease, and the loss of nourishment of meridians will lead to stroke [12, 13]. The symptoms of ACI are characterized by prominent pathogenic factors, and the treatment should comply with the principle of “treating the symptoms if it is acute and treating the root if it is chronic.” Because the basic pathogenesis is that phlegm-heat causing wind and phlegm-blood accumulation, resulting in inversion of Qi and blood. The disease can be treated by the method of reviving the spirit with strengthening the body resistance as the primary task and dispelling wind and removing stasis as the secondary task [14]. The prescription group of Fuyuan Xingshen Decoction consists of *Codonopsis pilosula*, motherwort, *Acorus tatarinowii*, *Panax notoginseng*, leech, rhubarb, and Rhizomaarisaematis. *Codonopsis pilosula* can replenish Qi and strengthen the spleen and stomach. It is a fundamental medicine. *Panax notoginseng* can stop bleeding and expel stasis. Motherwort can activate blood circulation. Rhubarb has the effects of clearing heat and detoxification and dredging the internal organs. When combined with *Panax notoginseng*, it can stop bleeding without leaving stasis. Rhizomaarisaematis can clear away heat and phlegm. The combined use of these medicines can complement Qi, stop bleeding, disperse blood stasis, and clear heat and phlegm. Previous studies have shown that Fuyuan Xingshen Decoction can protect the blood-brain barrier, relieve cerebral edema, promote the homing of neural stem cells, promote microvascular angiogenesis, and improve the blood supply of brain tissues [15]. Butylphthalide injection can exert anti-apoptosis; improve mitochondrial function, anti-inflammatory, and other effects through the blood-brain barrier; and ultimately improve the function of nerve cells. In the clinical treatment of ACI, butylphthalide sodium chloride injection has been widely used and shows remarkable effects [16,  17]. In this study, Fuyuan Xingshen Decoction combined with butylphthalide sodium chloride injection was given to the observation group to observe the clinical effect.

RETRACTED

In this work, the observation group exhibited a 90.48% effective rate which was considerably higher than the control group (71.43%). Compared with the control group, the improvement in NIHSS, Barthel index, Mini-cog, and MoCA scores was larger in the observation group after treatment. The improvement degree of Vp, PI, Vm, and other hemodynamic indices was greater than the control group. This indicates that Fuyuan Xingshen Decoction combined with butylphthalide sodium chloride injection had good efficacy in ACI treatment and can effectively improve the cerebral nerve function, daily living ability, cognitive function, and cerebral hemodynamics of patients. Previous investigations have demonstrated that butylphthalide injection can efficiently improve cerebral nerve function in patients with cerebral infarction [18]. In addition, the drug can promote cerebrovascular neovascularization; improve the circulation of ischemic brain tissue; increase collateral blood flow in the infarct area; and ultimately reduce the nerve injury of patients and improve the degree of neurological impairment, daily living ability, cognitive function, and hemodynamics [19]. Fuyuan Xingshen Decoction can promote cerebrovascular neovascularization with the improved blood supply of brain tissue. The combination of the two drugs played a synergistic effect and further improved the cerebral nerve function and cerebral blood flow state of ACI patients [20].

The pathogenesis of ACI involves inflammatory response, atherosclerosis, extracellular matrix reconstruction, and other mechanisms. Its basic pathological mechanism is cerebral ischemia and hypoxia-related nerve tissue injury. UCH L1 is a specific neuronal protein product that can deubiquitinate and stabilize intracellular ubiquitin monomers and participate in cell proliferation, differentiation, and apoptosis. According to Liu and Ho [21], the level of UCH-L1 expression in serum was significantly higher in ACI patients than in healthy volunteers, and its expression level was favorably associated with the cerebral infarction size and the degree of neurological impairment. Fibulin-5, a glycoprotein, is secreted by a variety of vascular cells including fibroblasts, endothelial cells, and vascular smooth muscle cells. Fibulin-5, via binding to integrin, can enhance extracellular matrix adherence to endothelial cells and have a protective role in the blood-brain barrier [22]. It has been shown that the level of Fibulin-5 expression is dramatically elevated in the serum of ACI patients, and its level is favorably associated with the cerebral infarction size and the degree of neurological impairment [23]. VILIP-1 is a small molecule cytoplasmic protein with high nervous system specificity mainly expressed in neurons of the brain, can bind to calcium ions, and play a biological role in regulating calcium balance. According to relevant studies, VILIP-1 is found in significant concentrations in the serum of ACI patients, and the level of serum VILIP-1 can be used to evaluate the incidence of cerebral infarction and is closely associated with the progression of brain injury [24]. In this investigation, lower serum levels of UCH-L1, Fibulin-5, and VILIP-1 were observed in the observation group following treatment than in the control group, indicating that Fuyuan Xingshen Decoction in combination with butylphthalide injection can efficiently control the biochemical markers of neurological dysfunction in ACI patients. This could be associated with its effect on improving cerebrovascular microcirculation and inhibiting inflammatory response, and its exact mechanism must be investigated further.

miRNA is one of the noncoding microRNAs, which can regulate target mRNA transcription and translation by binding to the 3′ non-translation region of target mRNA. Circulating miRNA has high stability. The development of modern medical technology also enables the current detection technology to detect miRNA accurately and quickly. miRNAs have become biomarkers for early diagnosis of disease. miR-34c mitigated the inflammatory response by regulating the apoptosis of MI-type microglia. Furthermore, miR-34c could also target the activation of NLRP3 inflammasome and play a role in improving neuralgia in mouse experiments [25]. miR-25 plays a certain regulatory role in non-small cell carcinoma, breast cancer, and other malignant tumor diseases. It has been shown that miR-25 levels in the peripheral blood of ACI patients are considerably lower than those of healthy controls [26]. According to findings from other basic investigations, miR-25 plays a protective role in cerebral ischemia-reperfusion injury [27]. miR-182 can aggravate brain injury by downregulating the expression of anti-apoptotic proteins and regulating the oxidative stress process, which is directly associated with the development and occurrence of cerebral infarction; and its relative expression level is significantly increased in the peripheral blood of ACI patients [28]. In this investigation, the level of miR-25 expression was found to be increased in the observation group as compared to the control group, while the expression levels of miR-34c and miR-182 were both determined to be decreased in the control group after being treated. These demonstrate that Fuyuan Xingshen Decoction in combination with butylphthalide injection had better efficacy in the treatment of ACI than butylphthalide injection alone, which can improve the molecular level of miRNA more effectively. No significant differences in the incidence of adverse reactions were observed between the groups. This suggests that the incorporation of Fuyuan Xingshen Decoction into the observation group did not increase the number of adverse reactions, demonstrating the safety of Fuyuan Xingshen Decoction.

RETRACTED

In conclusion, Fuyuan Xingshen Decoction combined with butylphthalide injection can effectively improve neurological impairment, daily living ability, cognitive ability, and cerebral hemodynamics in patients with ACI, with a good effect and clinical application value in ACI treatment. However, this study also has shortcomings such as small sample size and unclear molecular mechanism. In the future, the research sample can be further expanded and the specific mechanism can be explored to provide more support for clinical application.

## Figures and Tables

**Figure 1:** Comparative analysis of the UCH-L1 level before and after treatment between the groups.

**Figure 2:** Comparative analysis of the Fibulin-5 level before and after treatment between the groups.

**Figure 3:** Comparative analysis of the VILIP-1 level before and after treatment between the groups.

**Figure 4:** Comparative investigations of the miR-34c expression levels between the groups.

**Figure 5:** Comparative investigations of the miR-25 expression levels between the groups.

**Figure 6:** Comparative investigations of the miR-182 expression levels between the groups.

**Table 1:** Comparative analysis of the clinical efficacy of the two groups (cases (%)).

Group	Clinical recovery	Markedly effective	Effective	Ineffective	Total effective
Observation group (*n* = 42)	12 (28.57)	15 (35.71)	11 (26.19)	4 (9.52)	38 (90.48)
Control group (*n* = 42)	8 (19.05)	14 (33.33)	8 (19.05)	12 (28.57)	30 (71.43)
*χ* ^*2*^-value					4.941
*P* value					0.026

**Table 2:** Comparative analysis of NIHSS, Barthel index, Mini-cog, and MoCA scores between the groups before and after treatment ($\bar{x}\pm s$, points).

Group	NIHSS score		Barthel index score		Mini-cog score		MoCA score	
	Before treatment	After treatment	Before treatment	After treatment	Before treatment	After treatment	Before treatment	After treatment
Observation group (*n* = 42)	10.67 ± 3.05	5.26 ± 2.05^a^	47.85 ± 4.73	75.55 ± 8.85^a^	15.46 ± 2.09	27.24 ± 2.98^a^	16.29 ± 2.04	26.86 ± 2.44^a^
Control group (*n* = 42)	10.83 ± 3.48	8.26 ± 3.77^a^	46.98 ± 3.83	59.02 ± 4.78^a^	15.67 ± 3.11	21.99 ± 3.08^a^	15.76 ± 2.84	20.57 ± 2.86^a^
*t*-value	0.234	4.533	0.938	10.652	0.558	3.298	0.972	10.855
*P* value	0.816	<0.001	0.351	<0.001	0.992	<0.001	0.334	<0.001

*Note*. In contrast to before treatment, ^a^*P* < 0.05.

**Table 3:** Comparative analysis of the two groups' hemodynamic indices before and after treatment ($\bar{x}\pm s$, points).

Group	Vp (cm/s)		PI		Vm (cm/s)	
	Before treatment	After treatment	Before treatment	After treatment	Before treatment	After treatment
Observation group (*n* = 42)	56.35 ± 4.86	69.40 ± 6.00^a^	0.89 ± 0.05	0.60 ± 0.08^a^	26.82 ± 2.39	38.71 ± 3.24^a^
Control group (*n* = 42)	55.66 ± 5.56	62.87 ± 5.65^a^	0.89 ± 0.12	0.75 ± 0.10^a^	27.40 ± 2.16	32.11 ± 3.41^a^
*t*-value	0.603	5.132	0.048	7.168	1.166	9.083
*P* value	0.548	<0.001	0.962	<0.001	0.247	<0.001

*Note.* In contrast to before treatment, ^a^*P* < 0.05.

RETRACTED

**Table 4:** Comparative evaluation of serum levels of UCH-L1, Fibulin-5, and VILIP-1 between the groups before and after treatment ($\bar{x}\pm s$).

Group	UCH-L1 (ug/l)		Fibulin-5 (ug/l)		VILIP-1 (ug/l)	
	Before treatment	After treatment	Before treatment	After treatment	Before treatment	After treatment
Observation group (*n* = 42)	0.69 ± 0.40	0.28 ± 0.06^a^	91.32 ± 9.33	21.13 ± 3.71^a^	8.07 ± 2.28	2.05 ± 1.19^a^
Control group (*n* = 42)	0.64 ± 0.29	0.40 ± 0.22^a^	90.96 ± 9.25	57.27 ± 5.20^a^	8.32 ± 2.03	4.47 ± 1.91^a^
*t*-value	0.724	3.564	0.180	36.678	0.513	6.965
*P* value	0.471	0.001	0.858	<0.001	0.610	<0.001

*Note.* In contrast to before treatment, ^a^*P* < 0.05.

**Table 5:** Comparison of miR-34c, miR-25, and miR-182 expression levels in peripheral blood before and after treatment in the groups ($\bar{x}\pm s$).

Group	miR-34c		miR-25		miR-182	
	Before treatment	After treatment	Before treatment	After treatment	Before treatment	After treatment
Observation group (*n* = 42)	1.19 ± 0.05	0.73 ± 0.07^a^	0.63 ± 0.12	0.95 ± 0.17^a^	2.72 ± 0.77	1.18 ± 0.53^a^
Control group (*n* = 42)	1.18 ± 0.07	0.98 ± 0.07^a^	0.63 ± 0.09	0.78 ± 0.09^a^	2.78 ± 0.68	2.09 ± 0.62^a^
*t*-value	0.324	15.706	0.072	5.630	0.364	7.184
*P* value	0.747	<0.001	0.943	<0.001	0.717	<0.001

*Note*. In contrast to before treatment, ^a^*P* < 0.05.

**Table 6:** Comparative analysis of adverse reactions between the groups (cases (%)).

Group	Abdominal discomfort	Fever	Nausea	Headache	Dry throat	Total adverse reaction rate
Observation group (*n* = 42)	1 (2.38)	1 (2.38)	1 (2.38)	1 (2.38)	1 (2.38)	5 (11.90)
Control group (*n* = 42)	0 (0.00)	1 (2.38)	0 (0.00)	2 (4.76)	0 (0.00)	3 (7.14)
Fisher's exact probability value						0.713

## Data Availability

The labeled dataset that supports the findings of this study is available from the corresponding author upon request.
